The article "Expanded alleles of the FMR1 gene are related to unexplained recurrent miscarriages" was retracted in 2019. Reason: concerns about the data.

# Expanded alleles of the *FMR1* gene are related to unexplained recurrent miscarriages

**DOI:** 10.1042/BSR20170856

**Published:** 2017-11-23

**Authors:** Xin-hua Wang, Xiao-hua Song, Yan-lin Wang, Xing-hua Diao, Tong Li, Qing-chun Li, Xiang-hui Zhang, Xiao-hui Deng

**Affiliations:** 1 Department of Reproductive Medical Center, Qilu Hospital, Shandong University, Jinan, Shandong 250012, China; 2 Department of Reproductive Medicine, Affiliated Hospital of Binzhou Medical College, Binzhou, Shandong 256603, China; 3 Department of Obstetrics and Gynecology, Binzhou People’s Hospital, Binzhou, Shandong 256610, China; 4 Xinshijie Zhongxing Eye Hospital, Shanghai 200050, China

**Keywords:** abortions, FMR1 expanded alleles, fragile X premutations, intermediate zone carriers, unexplained recurrent miscarriages

## Abstract

Up to 50% of recurrent miscarriage cases in women occur without an underlying etiology. In the current prospective case–control study, we determined the impact of CGG trinucleotide expansions of the fragile-X mental retardation 1 (*FMR1*) gene in 49 women with unexplained recurrent miscarriages. Case group consisted of women with two or more unexplained consecutive miscarriages. Blood samples were obtained and checked for the presence of expanded alleles of the *FMR1* gene using PCR. Patients harboring the expanded allele, with a threshold set to 40 repeats, were further evaluated by sequencing. The number of abortions each woman had, was not associated with her respective CGG repeat number (*P*=0.255). The repeat sizes of CGG expansion in the *FMR1* gene were significantly different in the two population groups (*P*=0.027). All the positive cases involved intermediate zone carriers. Hence, the CGG expanded allele of the *FMR1* gene might be associated with unexplained multiple miscarriages; whether such an association is coincidental or causal can be confirmed by future studies using a larger patient cohort.

## Introduction

Involuntary loss of pregnancy in the first 24 weeks before the fetus is viable is termed as miscarriage. Recurrent miscarriage is defined as three or more consecutive pregnancy losses and is seen in 1% of women becoming pregnant [1–3]. There are multiple causes of recurrent miscarriage, involving genetic predisposition, anatomical, infectious, immunological, hematological, and endocrinology-related factors. However, etiology is unknown in 50% of recurrent miscarriage cases [4].

The fragile-X mental retardation 1 (*FMR1*) gene is located in the X chromosome, and encodes the fragile-X mental retardation protein (FMRP), an RNA-binding protein that regulates translation by regulating mRNA export between the cytoplasm and nucleus [5]. FMRP is required for normal neural development. *FMR1* gene mutations involve an expansion of CGG trinucleotide repeat region in the 5′-UTR [5] of *FMR1* mRNA. Fragile-X syndrome, premature ovarian failure (POF), and fragile X-associated tremor-ataxia syndrome (FXTAS) are different diseases associated with CGG expansion and each one is characterized by a different degree of this expansion [6].

The article "Expanded alleles of the FMR1 gene are related to unexplained recurrent miscarriages" was retracted in 2019. Reason: concerns about the data.

Normal people carry up to 54 CGG repeats, while full mutation refers to more than 200 repeats. An expansion from 55 to 200 is called premutation, while the presence of 41–54 repeats is termed as the ‘gray’ or intermediate zone [7,8]. The prevalence of premutation is approximately 1 to 250 women [9], which can reach up to 1 to 110 in specific populations [10]. The intermediate zone can be found in 1 to 57 women [11]. Premutation with 55–200 CGG repeats has been shown to be related to POF [12]. Hence, the objective of the current study was to determine if CGG repeat expansion is associated with the risk of miscarriage.

## Methods

### Patients

The study was approved by the Institutional Review Board of Affiliated Hospital of Binzhou Medical College, and was conducted in accordance with the Declaration of Helsinki. The study population was recruited between 1 January 2014 and 31 December 2016 from recurrent miscarriage outpatient clinic of Affiliated Hospital of Binzhou Medical College of China. Inclusion and exclusion criteria are summarized in Table 1. The inclusion and exclusion criteria were stringent to minimize the risk of bias, a problem inherent in retrospective studies. Data from their medical records were obtained and additional laboratory examinations were ordered, when needed. The control group consisted of women from the outpatient gynecological clinic at the Affiliated Hospital of Binzhou Medical College of China, visiting for routine diagnostic checkup, as well as female members of hospital staff, age matched within 2 years, on a 1:1 ratio. Recurrent miscarriage in the present study was considered the presence of at least two consecutive pregnancy losses.

**Table 1:** Inclusion and exclusion criteria used in the current study

**Inclusion criteria**
Cases
Age at recruitment <40 years Two or more consecutive pregnancy losses up to completion of 20 weeks of pregnancy (with/without prior successful pregnancy)
Controls
Age at recruitment <40 years History of documented normal pregnancies
**Exclusion criteria**
Cases
History of abortion due to infection (TORCH, syphilis, HBV, HCV, HIV) Currently in pregnancy or puerperium (6-week postpartum) Diagnosis of thrombophilia (hereditary or acquired) History of deep vein thrombosis or pulmonary Diagnosed anatomical abnormalities of the uterus or fallopian tubes (including submucosal fibroids, uterine septum, Asherman syndrome) History of cervical insufficiency History of surgical procedures in the pelvis (excluding cesarean section) History of alcohol/drug abuse History of cancer Abnormal chromosomal karyotype (in the couple) Abnormal controls History of pregnancy loss Use of assisted reproduction technology

TORCH=toxoplasma gondii, rubella virus, cytomegalovirus herpes simplex virus; HBV=hepatitis B virus; HCV=hepatitis C virus

The article "Expanded alleles of the FMR1 gene are related to unexplained recurrent miscarriages" was retracted in 2019. Reason: concerns about the data.

### PCR analysis

Genomic DNA was isolated from peripheral blood leukocytes using an affinity purification method following manufacturer’s recommendation (Thermo Fisher Scientific, Shanghai, China). Genomic DNA samples were tested for the presence of an expansion in the CGG trinucleotide repeat region using a two-step PCR protocol [13]. In the first step, genomic DNA was amplified using PCR, with the following primers: forward: 5′- GCTCAGCTCCGTTTCGGTTTCACTTCCGGT-3′ and reverse: 5′-AGCCCCGCACTTCCACCACCAGCTCCTCCA-3′, a primer pair that flanks the CGG repeat region, using betaine as the osmolite14 and the Expand Long Template PCR System from Roche Diagnostics. The reaction mixtures were 500 μmol/l dNTPs, 0.20 μM of each primer, 50 ng of genomic DNA, and 2.2 M betaine.

The final PCR products were resolved by electrophoresis in 2.5% agarose gel in the presence of Ethidium Bromide for 1 h at 40 V. The expected PCR product with this method was 221 bp, excluding the CGG repeat region. The cutoff for identification of the positive cases was set at 41 repeats. Thus, the presence of a band between 344 and 383 bp defined ‘the gray zone’, while a band between 384 and 821 bp the ‘premutation state’. Gel analysis was performed using Image Lab software (Bio–Rad). The results marked as positive were verified with sequencing analysis to confirm the length of the expanded alleles. All PCR reactions that produced a single band were subsequently analyzed with the second PCR step, using the reverse primer mentioned above and the CGG-chimeric primer (5′- AGCGTCTACTGTCTCGGCACTTGCCCGCCGCCGCCG-3′), under the same conditions. Of note, the 3′ end sequence of the chimeric primer (CCGCCGCCGCCG) has the potential to bind randomly in the CGG repeat region, and thus to produce a ‘smear’ on the gel, in the presence of expanded mutated alleles that were not amplified in the first step [14].

### Sequencing analysis

All PCR fragments, from the specimens that were considered as positive, were gel isolated, purified, and further analyzed by dideoxy-termination sequencing method performed by a locally available sequencing core to accurately measure the number of the repeats.

The article "Expanded alleles of the FMR1 gene are related to unexplained recurrent miscarriages" was retracted in 2019. Reason: concerns about the data.

### Statistical analysis

Statistical analysis was performed using IBM SPSS Statistics v21. Continuous data were described either as median or mean ± S.D. – frequencies as *n* (%). Comparison between groups in continuous variables was performed using Mann–Whitney test and comparison amongst more than two groups was performed using the Kruskal–Wallis test. A model of linear regression was created, for predicting values, after accurately measuring a number of them by sequencing. Significance level was set to 0.05.

## Results

Following screening process as mentioned in the inclusion criteria, a total of 57 cases were selected and another 57 controls were recruited, age matched (within ±2 years). The major characteristics of the study population and the main results are summarized in Table 2. The women in the patient group had two up to five miscarriages (average 2.52 ± 0.63). The percentage of women with two miscarriages was 59.6%, with three miscarriages 29.8%, with four miscarriages 8.8%, and with five miscarriages 1.8% (Table 3). The number of miscarriages each woman had was not associated with the number of the CGG repeats (Kruskal–Wallis test, *P*=0.255).

**Table 2:** Summary characteristics and results in the study population

	Cases	Controls	*P*-value
*n*	57	57	
Age (years)	33 (28–39)	33 (29–38)	0.906
Miscarriages	2.52 ± 0.63	–	
Women with three or more miscarriages	23 (40%)		
CGG repeats*	35 (31–38)	31 (30–33)	0.017
CGG repeats^†^	29 (26–31)	28 (25–28)	0.027
Intermediate zone	4	1	0.168
(41–54 CGG repeats)			
Odds ratio: 4.167			

Continuous variables are presented as median (25–75th percentile) or mean ± S.D. and dichotomous variables as *n* (%); * estimated by electrophoresis analysis; ^†^ calculated by linear regression analysis.

**Table 3:** Distribution number (#) of miscarriages in the included study population

# of miscarriages	Cases	% of cases group
2	34	59.6
3	17	29.8
4	5	8.8
5	1	1.8
	**57**	**100**

Analysis of the first PCR step amplicons revealed a distinct, two band patterns in 34 out of 57 of patients and 22 out of 57 of control samples (Figure 1, representative figure). The samples that showed a ‘single band’ were further analyzed with the second PCR step to distinguish homozygosity, from the presence of a mutated allele not amplified in the first step. No mutated allele was detected. For each woman in the study, the band representing the highest number of CGG repeats was taken into account.

**Figure 1:** Representative gel electrophoresis analysis of PCR products Shown are different repeat numbers.

Five women from the patients group (7.01%) were identified to carry the expanded allele – 46, 50, 55, 58, and 65 repeats (two intermediate zone and three premutation carriers), while only one woman in the control group (1.75%) was identified to carry an expanded allele with 57 repeats (premutation). The reported prevalence of intermediate zone carriers is up to approximately 1/57 (1.75%) as mentioned before. The two groups do not differ in terms of number of women marked positive for premutation (Chi-square, *P*=0.168, odds ratio =4.167, ci 0.459–39.629). The number of repeats of the two population groups were significantly different (Mann–Whitney test, *P*=0.027).

The article "Expanded alleles of the FMR1 gene are related to unexplained recurrent miscarriages" was retracted in 2019. Reason: concerns about the data.

In order to determine the exact number of repeats present in each allele, the positive cases were evaluated by sequencing. Except for one case within the miscarriage group, all the remaining five had intermediate zone CGG expansion, extending from 42 to 47 repeats (Table 4).

**Table 4:** Measured number (*n*) of CGG repeats using electrophoresis compared with sequencing analysis, on cases marked as positive (one case was measured as normal, <41 repeats)

*n* of CGG repeats	**Cases**					**Controls**
**Electrophoresis**	46	50	55	58	65	57
**Sequencing analysis**	38	42	44	44	47	46

Even though electrophoresis results were largely consistent with sequencing analysis, PCR-based analysis did result in an overestimation in each case, with one out of six cases not getting validated by the sequencing analysis. A regression model in SPSS was used to plot divergence between the two methodologies and linear regression was found to be a good fit (Figure 2), which was then used for CGG repeat prediction in all 114 cases and controls in the current study (Table 5).

**Figure 2:** Linear regression analysis of electrophoresis compared with sequencing, as methods of measuring CGG repeats One out of six cases did not get validated by the sequencing analysis; hence there are 11 instead of 12 data points.

**Table 5:** Total number of CGG repeats including both bands after regression analysis

	Cases			Controls	
CASE ID *n*	**First band**	**Second band**	Controls ID *n*	**First band**	**Second band**
**1**	27	25	**101**	25	25
**2**	27	27	**102**	27	24
**3**	28	27	**103**	25	25
**4**	28	26	**104**	28	17
**5**	26	20	**105**	25	25
**6**	27	27	**106**	27	24
**7**	33	25	**107**	28	28
**8**	26	19	**108**	30	18
**9**	26	26	**109**	22	22
**10**	28	27	**110**	29	21
**11**	25	22	**111**	20	20
**12**	25	25	**112**	27	27
**13**	44	31	**113**	24	21
**14**	25	25	**114**	29	20
**15**	27	25	**115**	27	27
**16**	33	26	**116**	27	24
**17**	25	25	**117**	27	27
**18**	29	29	**118**	27	27
**19**	33	30	**119**	25	25
**20**	35	22	**120**	27	25
**21**	47	38	**121**	24	24
**22**	38	34	**122**	25	25
**23**	20	20	**123**	27	20
**24**	26	24	**124**	29	20
**25**	25	25	**125**	27	27
**26**	25	23	**126**	29	22
**27**	32	17	**127**	26	26
**28**	44	15	**128**	26	23
**29**	30	28	**129**	25	25
**30**	19	19	**130**	32	28
**31**	26	19	**131**	28	28
**32**	28	20	**132**	27	24
**33**	30	20	**133**	26	26
**34**	42	27	**134**	20	20
**35**	35	33	**135**	28	26
**36**	28	20	**136**	31	24
**37**	28	20	**137**	23	23
**38**	32	28	**138**	24	24
**39**	29	28	**139**	29	20
**40**	26	26	**140**	27	27
**41**	25	25	**141**	28	28
**42**	27	25	**142**	46	22
**43**	28	28	**143**	27	27
**44**	29	19	**144**	27	20
**45**	30	25	**145**	24	24
**46**	31	26	**146**	27	24
**47**	24	24	**147**	22	22
**48**	24	24	**148**	29	20
**49**	30	19	**149**	20	20
**50**	28	20	**150**	29	29
**51**	21	21	**151**	23	19
**52**	32	24	**152**	25	20
**53**	32	25	**153**	28	23
**54**	29	23	**154**	26	22
**55**	31	25	**155**	25	19
**56**	28	28	**156**	24	23
**57**	27	23	**157**	25	21

Underline represents the positive cases (four in cases and one control).

The article "Expanded alleles of the FMR1 gene are related to unexplained recurrent miscarriages" was retracted in 2019. Reason: concerns about the data.

## Discussion

In the present study, we examine the presence of expanded CGG alleles in women with unexplained recurrent miscarriages. These women have significantly more CGG repeats at their *FMR1* gene, than women with documented normal fertility.

It is well known that women with premutations of the *FMR1* gene are likely to develop POF in up to 20% of cases [15]. On the contrary, women with intermediate length alleles do not seem to carry this risk [16]. Since none of the women in this study had a premutation of the *FMR1* gene, we cannot attribute the number of miscarriages directly to POF.

FMR1 alleles with the size of 45 to 200 are meiotic unstable and can be inherited as such or with increased size in the offspring [17], and also the *FMR1* gene undergoes abnormal methylation [18,19]. It is possible that these unstable mutations can result in defects that are incompatible with life, and lead to miscarriage. This could be proven by performing DNA analysis in the products of conception, in women with recurrent miscarriages, looking for expanded alleles or an otherwise altered *FMR1* gene (e.g. methylation).

The mechanism of meiotic instability of the *FMR1* gene occurs only during meiosis in oocytes and not in sperm [20]. Therefore, women with premutations can have daughters with full mutations, whereas men can only pass premutations to their daughters as such. So, it seems reasonable to focus screening to women, when examining couples for expanded CGG alleles.

The present study has its own limitations. As it is a case–control study, it is vulnerable to bias. Also, secondary causes of recurrent miscarriages have potential confounding effects and cannot be ruled out. Recurrent miscarriages are a cause of significant distress for the affected couples, and pose a diagnostic and therapeutic challenge for the physicians involved. This is especially true for the cases that remain unexplained, after the full diagnostic workup (approximately 50%). It is possible that the presence of a CGG expanded allele could explain a number of them. To our knowledge, there is no other similar study in the medical literature. More studies are needed toward this hypothesis in the future, which could verify it, and uncover the molecular mechanism responsible.

The article "Expanded alleles of the FMR1 gene are related to unexplained recurrent miscarriages" was retracted in 2019. Reason: concerns about the data.

## Abbreviations

CI: confidence interval
*FMR1*: fragile-X mental retardation 1
FMRP: fragile X mental retardation protein
FXTAS: fragile-X associated tremor-ataxia syndrome
POF: premature ovarian failure
